The article "An Efficient Model for Lungs Nodule Classification Using Supervised Learning Technique" was retracted in 2023. Reasons: signs of a paper mill; compromised peer review; unreliable results or conclusions.

# An Efficient Model for Lungs Nodule Classification Using Supervised Learning Technique

**DOI:** 10.1155/2023/8262741

**Published:** 2023-02-04

**Authors:** Fayez Eid Alazemi, Babar Jehangir, Muhammad Imran, Oh-Young Song, Tehmina Karamat

**Affiliations:** ^1^Department of Computer Science and Information Systems, College of Business Studies, The Public Authority for Applied Education & Training, Adailiyah 12062, Kuwait; ^2^Department of Computer Science & Software Engineering, Shaheed Zulfiqar Ali Bhutto Institute of Science & Technology, Islamabad, Pakistan; ^3^Software Department, Sejong University, Seoul, Republic of Korea; ^4^Department of Software Engineering, Foundation University Islamabad, Islamabad, Pakistan

## Abstract

Lung cancer has the highest death rate of any other cancer in the world. Detecting lung cancer early can increase a patient's survival rate. The corresponding work presents the method for improving the computer-aided detection (CAD) of nodules present in the lung area in computed tomography (CT) images. The main aim was to get an overview of the latest tools and technologies used: acquisition, storage, segmentation, classification, processing, and analysis of biomedical data. After the analysis, a model is proposed consisting of three main steps. In the first step, threshold values and component labeling of 3D components were used to segment the lung volume. In the second step, candidate nodules are identified and segmented with an optimal threshold value and rule-based trimming. It also selects 2D and 3D features from the candidate segmented node. In the final step, the selected features are used to train the SVM and classify the nodes and classify the non-nodes. To assess the performance of the proposed framework, experiments were performed on the LIDC data set. As a result, it was observed that the number of false positives in the nodule candidate was reduced to 4 FP per scan with a sensitivity of 95%.

## 1. Introduction

### 1.1. Significance of Study

In the current era, health care is an important domain in which a lot of research work has been carried out, various researchers working in the healthcare domain to solve the problems of healthcare applications, Sultan et al. [1] introduced a hybrid approach for Alzheimer patients through video summarization. Another research work in the health care domain is carried out by Bacanin et al. [2]; the authors used wireless sensing network technology to monitor human health, pollution predictions, and some other related factor that are useful for human health. Artificial Intelligence and machine learning techniques are very commonly used in the health care sector and researchers get very good results. An artificial intelligence-based technique by Chang et al. [3] was introduced; they offer a drug selection framework for the individualized selection of NSCLC patients using an artificial intelligence-assisted medical system. The method forecasts drug effectiveness-cost under the concept of ensuring efficacy while taking the economic cost of targeted drugs into account as an auxiliary decision-making element. Similarly Ramzan et al. [4] introduce a protection system for medical images; the author proposed a technique in which they secure medical images. Another medical base Optimal feature extraction and ulcer classification from WCE image data using deep-learning technique in introduced by [5] and another medical image-related work has been carried out by Azam et al. [6] which is also related to health care domain. So, lot of studies have been continuing in the health care domain. In the proposed research study we are also focusing on health care and specifically on lung cancer.

The article "An Efficient Model for Lungs Nodule Classification Using Supervised Learning Technique" was retracted in 2023. Reasons: signs of a paper mill; compromised peer review; unreliable results or conclusions.

Cancer is defined as abnormal cell development in tissues that disrupts the normal functioning of a human organ and, in severe circumstances, can result in death. Today, 100 different cancers have been reported, including bladder, breast, lung, skin, and thyroid cancer. In 2008, the American Cancer Society estimated that lung cancer was responsible for roughly 29% of all fatalities in the United States. In 2016, 1.6 million lung cancer cases were reported, with an estimated 60 thousand deaths. Lung cancer is now one of the leading causes of death in the United States. Among the three most fatal cancers, lung cancer kills more people than colon, breast, and pancreatic cancer [7]. Lung cancer may be identified at an earlier stage of the disease when it is more durable. The application of machine learning in medical image detection [8, 9] has increased in recent years, with the development of computer vision [10, 11] and artificial intelligence, among which machine learning is used in lung nodule detection the target detection network in deep learning [12, 13] can accurately locate the location of the region of interest and return its category.

In the proposed CAD scheme, there are three major steps involved, Lung volumes are segmented in the first stage using thresholding, which implies low-density and high-density regions are segregated from one another. Lung masks are then created by applying 3D-connected components labeling on the segmented image. After that, the mask was adjusted to remove noise and small holes while keeping the image's intensity. In the second step, rule-based pruning is used to detect and segment nodule candidates. Optimal multiple thresholding, i.e., the Otsu thresholding approach was applied to a segmented lung volume. Finally, in the last stage, nodule candidates are used to generating features' and are employed as a classifier.

The article "An Efficient Model for Lungs Nodule Classification Using Supervised Learning Technique" was retracted in 2023. Reasons: signs of a paper mill; compromised peer review; unreliable results or conclusions.

### 1.2. Lungs Nodule

The lung nodule is a development in the lung region that is oval or tiny and rounded in shape. It could be a “spot on the lung” or a “coin lesion” at times. The size of a nodule is usually between 0.5 and 3 cm; however, it can be greater. These nodules are usually caused by inflammation in the lungs. Inflammation can be caused by illness or infection. Noncancerous nodules commonly do not require remedy. If the nodules size is greater than 3 cm this would be more likely lung cancer is caused mostly by poor food quality, smoking, medications, and environmental pollution. Computerized image analysis now aids in the early detection of lung cancer, which includes the detection and classification of suspicious nodules.

There are two main reasons for lung cancer, first, it is very difficult to diagnose it at the early stages due to insufficiency of symptoms, and second, poor prognostics when the infection is detected more near the beginning phase. However, it is hard to diagnose early whether pulmonary nodules exist or not, and whether this nodule is a malignancy or not because the diagnosis system is not efficient. When radiologists diagnose one patient, they need to analyze computed tomography (CT) images with the naked eye. This existing system can be easy to mistake the diagnosis.

### 1.3. Computer-Aided Diagnostic

Computer-aided diagnostic (CAD) has been based on finding made by radiologists who explained the computer output based on quantitative analysis of radiological images. Textural highlights are essential for extracting features from a medical image. They provide information regarding spatial tonal variations and object surfaces. Descriptors are used successfully to advance the accuracy of the diagnosis system by picking noticeable features [14]. The basic idea in CAD schemes consists of four steps: the first one is the processing of images for extraction and detection of nodule candidates from the images, the second one is the image feature's quantization for candidates of abnormalities, the third one is a classification of data which differentiate between abnormal and normal features of lungs images (or benign and malignant), and the fourth and last one is quantitative assessment and recovery of pictures like those of obscure sores. In the lungs, tumor computer tomography (CT) is a standout among the most responsive method of detecting lungs nodule. A figured tomography (CT) sweep is an imaging technique that uses *X*-beams to take pictures of the cross-area of the body. An important point that needs to be considered is that the radiologist analysis is mainly based on the morphological structures under investigation which can be checked in 3D space and the examination of a CT is performed through bidimensional pictures that is why the tradeoff between the radiologists' needs to watch and what it appeared to him requires a remaking of the tridimensional parts of the tissue under investigation undertaking which other than intricate and moderate and during this reconstruction process lots of chances for mistakes.

The article "An Efficient Model for Lungs Nodule Classification Using Supervised Learning Technique" was retracted in 2023. Reasons: signs of a paper mill; compromised peer review; unreliable results or conclusions.

## 2. Literature Review

Over the past decades, various ideas and techniques have been proposed for the effective detection and classification of lung nodule detection.

Kuruvilla and Gunavathi [15] present a computer-aided classification using an artificial neural network for lung CT images. Lung images are converted into binary images by using a threshold selected from the Otsu method which is presented by Nobuyuki Otsu in 1979. Lung segmentation is carried out by using morphological operations. The author used statistical parameters like mean, standard deviation, and skewness for the classification of objects. The classification process is performed with the help of feed-forward (FF) and feed-forward back (FFB) propagation neural networks. The maximum classification accuracy of 91.1% has been achieved through the training function gradient descent backpropagation (training) network. The author proposed two new training functions based on existing ones, which give an accuracy of 93.3%.

Murphy et al. [16] evaluate thoracic CT scans for the automatic detection of nodules. In the preprocessing stage, the author firstly down-sampled the data so that an algorithm's speed can be increased. The full image contains 512 × 512-pixel values, converting that image to 256 × 256 pixels by block averaging. The author developed an algorithm by using the shape index (SI) and curvedness (CV) features of local images so that the initial candidate structure can be detected in the lung volume. SI and CV are used to establish the threshold and all voxels which lie between this range are considered seed points. Seed points are expanded based on hysteresis thresholding to form clusters. Clusters inside three voxels claiming one another are recursively consolidated until no more merging can be possible. After merging, discard the small clusters. After clustering, to ensure that candidates reside locally at the brighter spots, locations were initially checked and then adjusted. After that author applies two successive *k*-nearest neighbor classifiers in the reduction of false positives. After applying KNN classifications 90% true nodule.

The article "An Efficient Model for Lungs Nodule Classification Using Supervised Learning Technique" was retracted in 2023. Reasons: signs of a paper mill; compromised peer review; unreliable results or conclusions.

Shen et al. [17] discussed the problems that exist in the present methods, i.e., juxta-pleural nodules on lung boundaries are not fully addressed. To address this issue, author presents a computer-aided classification using a bidirectional coding method along with an SVM classifier to avoid oversegmentation and for smooth boundaries. The proposed system does not require any parameter to adjust. The authors first perform preprocessing to generate the initial mask using the Otsu adaptive thresholding technique; afterward, author-produced lung lobe masks by combining the flood filling method with 3D labeling. After segmentation author applies the bidirectional differential chain (BDC) method to detect both vertical and horizontal critical points. This helps in identifying inflection points. Inflection points are those where the boundary of convexity changes. For inflection point detection on a horizontal surface, first boundary pixels are generated from the lung boundary mask and then boundary encoding has been applied using horizontal codeword generation, arrow map generation, and codeword assignments. Similar steps were applied for the detection of inflection points in the vertical direction. Code words are smoothened by using the Gaussian low pass filter's uses 3 features to select critical points which include: boundary segmentation concave degree, relative boundary distance, and relative position distance. The authors used a 3-order polynomial kernel for classification. The 10-foldcross-validation has been used to access modal performance.

Javaid et al. [18] have defined that thickness and percentage wall connectivity are the basis for six groups of potential nodules. This study improves the computational time from 11 secs to 3.8 secs. Following are the steps mentioned in the study: input chest CT scan to the CAD system. Then, contrast enhancement was performed in the preprocessing stage. Lung region extraction from thorax using thresholding and morphological closing. Nodule detection and segmentation using *k*-mean clustering and morphological opening. The overall system sensitivity, specificity, accuracy, and FPs per scan are 91.65%, 96.67%, 96.22%, and 3.19FPs, respectively.

Wang et al. [19] have advised some new features which helped to reduce the number of FPs with better sensitivity. After the features were selected based on the convolution neural network (CNN) model learning from the nonmedical data especially data which lacks ground truth. Principal component analysis (PCA) is used to suppress ribs and improve lung nodule visibility. The lung is segmented based on the active shape model (ACM). Candidate nodule was retrieved through generalized Laplacian of Gaussian method (gLog). Features were extracted from handcrafted and deep-learning method. Finally, the cost-sensitive random forest (CS-RF) was trained to classify the lung nodule.

The article "An Efficient Model for Lungs Nodule Classification Using Supervised Learning Technique" was retracted in 2023. Reasons: signs of a paper mill; compromised peer review; unreliable results or conclusions.

Setio et al. [20] present multiview convolution networks in which nodule candidates are obtained by combining three candidate detectors specifically designed for solid, subsolid, and large nodules to automatically discriminate features from training data. The proposed architecture consists of various streams of 2D Convolution Networks, in which we can get the final classification by combining the outputs, using the dedicated fusion method. At 1 and 4 FPs per scan, the method has sensitivities of 85.4% and 90.1%.

Froz et al. [21] use texture features to separate nodules and non-nodules. For texture measurements, an artificial crawler (AC), rose diagram (RD), and a combination of AC and RD are used. AC and RD were built and applied before on 2D images. AC's and RD models are used as a base for the hybrid model. Feature vectors of these two models combine to form a single feature vector of the hybrid model. In the end, classification is carried out by using SVM. The system has been validated by accuracy, specificity, sensitivity, the variation coefficient of accuracy, and the receiver operating characteristic (ROC) curve.

Wang et al. [22] said that nodule segmentation is difficult if we have a diversity of lung nodules with similar visual aspects between nodules and their surroundings. This technique uses multiple branch CNN which simultaneously selects two types of features i.e., multiview 3D and local texture features. To extract features without using multiple networks author combines multiscale sections with multichannel sections. Features of the patch center are retained instead of the patch edge by the central pooling layer. During model training for an efficient model, sampling was carried out on imbalanced training labels and extracting challenging patches. In this strategy, weights are assigned to each voxel denoting its difficulty for segmentation. Through CF-CNN, the overall lung nodule segmentation performance has been improved especially for juxta plueral nodules. This does not depend on nodule shape or user-specified parameters.

Wang et al. [23] present multicrop convolutional neural network (MC-CNN) for an end-to-end computation by utilizing CNN. This method helps in feature extraction of high-level nodule malignancy classification. The proposed method does not use handcrafted-aided engineering and nodule segmentation. These methods are quite complex, time-consuming, and do not consider different types of nodules. A specialized pooling strategy i.e., multicrop pooling operation used to generate multiscale features so that the conventional max-pooling operation can be replaced. Instead of using multiple networks, the proposed approach provides better results when applied to a single network with less computational complexity. Estimation of nodule diameter and quantification of nodule semantic labels greatly helps to evaluate the malignancy uncertainty.

The article "An Efficient Model for Lungs Nodule Classification Using Supervised Learning Technique" was retracted in 2023. Reasons: signs of a paper mill; compromised peer review; unreliable results or conclusions.

Tajbakhsh and Suzuki [24] provide a comparison between end-to-end learning architectures. End-to-end machine learning eliminates the need for handcrafted features and provides a direct mapping of input to the finer output. The two end-to-end architectures are massive training artificial neural networks (MTANNs) and convolutional neural networks (CNNs). The function of MTANNs is to detect the focal lesions and then classify the as lesions. The first step involved in designing the multiple ANN image is to divide the nonlesion class into many subclasses and afterward train every MTANN to recognize the lesions and nonlesions. In computer vision, CNN gains much popularity in medical imaging in a short period. In the input image channel, the small subset of neurons is detected by convolutional layers. For detecting the same feature in the complete image the connection weight is shared between the nodes. Shared weights are called kernel or convolution kernel. To achieve the hierarchical features of an image and to minimize the computational cost, a pooling layer has been added between the convolutional layers.

Santos et al. [25] segment the structure present inside the lung by using Gaussian mixture models and hessian matrix. Shannon's and Tsallis's entropy are used for the calculation of texture descriptors whereas SVM is used for the classification of ROI as nodules and non-nodules. Hessian matrix is used for the separation of round structures that were separated from the blood vessels and bronchi. Small lung nodules are automatically detected by the presented study having a diameter ranging from 2 mm and 10 mm. This method indicates the presence of nodules but does not give information about exact boundaries.

Calle-Alonso et al. [26] presented the work for the classification of multiclass biomedical objects. In this method, a hybrid approach in combination with Bayesian regression and pairwise comparison, and the *k*-nearest neighbor technique is used. This method can be used in two possible ways i.e., fully automated way or a relevant feedback framework. In the relevant feedback framework, the data that is obtained by automatic classification, and experts are used to get the best results; here, learning stage is finished now and further classification can be carried out automatically. By using the same scheme as in the original studies, this method has been applied in the biomedical context.

The article "An Efficient Model for Lungs Nodule Classification Using Supervised Learning Technique" was retracted in 2023. Reasons: signs of a paper mill; compromised peer review; unreliable results or conclusions.

Messay et al. [27] have introduced a new algorithm for nodule segmentation, the author proposed three methods which include a fully automated (FA) that works on the principle of the TR segmentation engine, the second method is semiautomated system (SA) which employs TRE segmentation engine and the last method is a hybrid system which works by using both FA and SA systems. In the FA system, only one user is needed while in the SA system, 8 users supplied points are required. The hybrid system works by using the single-user feature of the FA system and good quality results of the SA system but if a single-user Cue point is not enough then 8 control points can be added.

Khatami et al. [28] presented the study work in which multiclass radiography images were classified by using the three-step framework. In the first step, the denoising technique is applied, based on wavelet transform (WT). Less important features of images and noise were removed by using the statistical Kolmogorov Smirnov (KS). In the second step, unlabeled features were learned with the help of the deep belief network (DBN). Small-scale DBNs are efficient in use but in the case of larger networks, it is not cost-effective. Noise in images can produce a negative impact on the output of DBNs. DBNs can be improved by the combination of WT and KS. The features which are outputs of the first two steps act as input into classifiers for evaluation. The data collected from the results show that by using this three-step procedure, we can reduce the cost and can get high performance for image classification. So the proposed study can be used in the medical field for the analysis of noisy images in the diagnosis of different diseases of skeleton, muscles, breast, and lungs.

Hussain et al. [29] have proposed a hybrid approach for lung nodule detection using a deformable model and distance transform. This proposed methodology has four major steps. In the first step, lung parenchymal and linear interpolation techniques are used to perform the lung segmentation, in the second step, multiple thresholding is used to extract ROI, and in the third step, the nodule is detected using a deformable model and distance transform. In the fourth and last step, fuzzy rule base pruning is used to reduce false positives.

Accurate lung segmentation has a direct impact on systems performance, but the problem identified in several approaches studied during the literature is that most of the techniques can extract the specific type of data and fails when slightly different input has been given. For example, when applying the region growing method on a high level of abnormality images then it fails during the segmentation stage, morphological operators can remove some important small nodules, and some methods ca not be able to include juxta-pleural nodules which lie across the boundaries.

The article "An Efficient Model for Lungs Nodule Classification Using Supervised Learning Technique" was retracted in 2023. Reasons: signs of a paper mill; compromised peer review; unreliable results or conclusions.

## 3. Proposed Model

The necessity sent of early detection of lung abnormalities has been emphasized by an automated lung nodule system. The proposed CAD system depicted in Figure 1 is a block diagram with three key components. Lung volumes are segmented in the first stage using thresholding, which implies low-density and high-density regions are segregated from one another. Lung masks are then created by applying 3D-connected components labeling on the segmented image. After that, the mask was adjusted to remove noise and small holes while keeping the image's intensity. Rule-based pruning is used to detect and segment nodule candidates in the second stage. To generate a region of interest (ROI), optimal multiple thresholding, i.e., the Otsu thresholding approach was applied to a segmented lung volume. Finally, nodule candidates are used to generate features' and are employed as a classifier in the last stage, with the primary goal of determining whether the nodule is malignant or benign.

### 3.1. Images Data Collection (Dataset)

The images of the lungs were obtained from the lung image database consortium (LIDC). Around 20 patients' data were obtained for this investigation, totaling over 4000 digital imaging and communications in medicine (DICOM images). DICOM is an international standard for transmitting, storing, retrieving, printing, processing, and displaying medical imaging data. In January 2000, CT-scan was used to obtain data from the patients. An original DICOM Lung image is shown in Figure 2(a). DICOM images provide detailed information about the image being taken, such as the date the image was acquired, the image's size, width, height, bit-depth, color type, and more.

### 3.2. Data Preprocessing

Sometimes images acquired from devices lack in comparison and brightness because of the restrictions of imaging substructures and illumination conditions also have an impact on the surrounding environment. At this point, image enhancement techniques have been used to make the image capable of appropriately capturing the features. For that noise filtering, contrast enhancement, and edge enhancement were performed to enhance the image. Figure 2(a) represents the original DICOM image and Figure 2(b) represents an enhanced image.

### 3.3. Lung Volume Segmentation

It is a crucial preprocessing step because it has a significant impact on the nodule detection result. The primary goal is to distinguish the lung cavity from the surrounding lung structure. Three steps can be taken to accomplish this: thresholding was used to obtain the first lung mask. The 3D volume is represented by *I* (*x*, *y*, *z*), where *x* and *y* are slice coordinates and *z* is the slice number. The volume is made up of several slices, each of which is the same size. High-density voxels depict the body around the lung cavity, while low-density voxels represent the lung cavity. To distinguish lung parenchyma from lung architecture, a fixed threshold was applied. After performing fixed thresholding, Figure 3(a) depicts the lung region. The initial lung capacity is calculated as follows:

(1) $$\begin{array}{c} Si\left(x,y,z\right)=I\left(x,y,z\right)<-500\text{.} \end{array}$$

In equation (1), Si is Shape Index and *I* is the 3D volume and *x* and *y* are the slice coordinates and *z* is the slice number. After thresholding, the black area represents body voxels and white represents nonbody voxels. For extracting the lung region within nonbody voxels of thresholded lung volume 3D-connected labeling was applied with 18 connected neighbors [3]. In response to that the labeled volumes L are obtained, from which the largest two volumes have been selected as lung region. In this way, unwanted components of the nonbody region are ignored during volume selection.

(2) $$\begin{array}{c} Si=\left.I_{first}\right|I_{second}\text{,} \end{array}$$

where *I* first represents the first largest volume and *I* second represents the second largest in labeled volume.  Figure 4(a) represents the two big lung volumes. After this stage, only small holes are left in the lung region which would be filled by applying a morphological hole-filling operation.  Figure 4(b) shows Lung volume after applying morphological operation.

The article "An Efficient Model for Lungs Nodule Classification Using Supervised Learning Technique" was retracted in 2023. Reasons: signs of a paper mill; compromised peer review; unreliable results or conclusions.

The lung mask does not have a juxta-pleural nodule in it, which influences systems performance. To include juxta-pleural nodules we use chain code analysis with eight angular directions: 0°, 45°, 90°, 135°, 180°, 225°, 270°, and 315°. After applying chain code, a Gaussian smoothing filter will be used for removing noise. By analyzing the transition critical points are used for the formation of the critical section. If the distance between two critical points is less than the nodule diameter then select it for critical section correction. After that fill in the critical section by joining critical points.  Figure 5(a) represents results after applying the chain code method with hole filling and Figure 5(b) represents the intersection of the original image with a segmented image to obtain a lung mask. Figures 6(a) and 6(b) represent the greyscale representation of the ROI.

### 3.4. Feature Extraction

It is a key element that describes nodules candidates. Nodule candidate detection is a key element, and the performance of automated systems relies heavily on nodule candidate selection. First ROI is extracted and then detected nodule candidates from segmented ROIs.

It is quite hard to extract ROIs because of the wide intensity range and multiple levels of vessel attachment. The researcher used to mean or fixed the values as base thresholds which sometimes fail to produce good results that is why we have used optimal threshold values. For calculating the optimal threshold, the median slice has been chosen because it contains the largest lung region, and the mean value of the pixel is calculated and used as the base threshold.  Figure 7(a) represents the ROI.

(3) $$\begin{array}{c} T^{\begin{array}{c} \left(i+1\right) \end{array}}=\frac{\mu_{0}+\mu_{b}}{2}\text{.} \end{array}$$

Rule-based pruning is required because when detecting nodule candidates through thresholding it may result in non-nodule. Vessels might be selected as nodule candidates. Thresholding may affect systems' accuracy and increase computational resource utilization. For avoiding this problem, rule-based pruning is applied on every ROI so that unnecessary non-nodules would be removed.  Figure 7(b) represents the ROI after applying rule-based pruning.

Four rules have been set for rule-based pruning. Rules are based on features of nodule candidates such as Area, Diameter, Volume, Circularity, and Elongation. Nodules are compared with a specific minimum and maximum threshold value and are removed from candidate nodules if they are below the threshold level.  Table 1 represents the pruning rules.

### 3.5. Nodule Detection

Nodules can be detected based on the feature vector, and from the feature vector, initial population would be generated. Based on the fitness function the system decides either to create a new generation with the help of genetic functions like crossover, mutation, and replication or that would be the one for which all the processing would happen. Later, SVM would be applied to find whether it is a malignant nodule or a benign nodule.  Figure 8 represents the steps from feature selection to classification.

### 3.6. Feature Selection

There are several possible features we can extract like geometric-based, statistical-based, texture-based, shape-based, etc., but most of the researchers used 2D- and 3D-based geometric features and 2D- and 3D-based statistical features. 2D Geometric features include area (*f*1), diameter (*f*2), perimeter (*f*3), and circularity (*f*4). 3D Geometric feature include volume (*f*5), compactness (*f*6), and elongation (*f*7). 2D intensity-based statistical feature consist of minimum (*f*8), mean (*f*9), variance (*f*10), skewness (*f*11), kurtosis (*f*12), and mean outside (*f*13) the segmented region. Features have been displayed in tabular format in Table 2.

The article "An Efficient Model for Lungs Nodule Classification Using Supervised Learning Technique" was retracted in 2023. Reasons: signs of a paper mill; compromised peer review; unreliable results or conclusions.

### 3.7. Performance Evaluation

To evaluate the data collected from LIDC [30], the classification capability of the nodule candidates depends on their sensitivity, specificity, accuracy, and false positives per scan.

### 3.8. Sensitivity

It measures the percentage of actual positives that are correctly recognized. This represents the percentage obtained from segmented slices containing cancerous nodules that are efficiently classified as cancerous.

(4) $$\begin{array}{c} \frac{TP}{\left(TP+FN\right)}\text{,} \end{array}$$

where TP is True Positives and FN is False Positives.

### 3.9. Specificity

It measures the percentage of negatives that are correctly recognized. This represents the percentage obtained from segmented slices containing cancerous nodules is efficiently classified as noncancerous.

(5) $$\begin{array}{c} \frac{TN}{\left(TN+FP\right)}\text{.} \end{array}$$

### 3.10. Accuracy

A statistical measure represents, how efficiently a classifier classifies a condition. The accuracy is the proportion of true results (both TP and TN) in the given dataset.

(6) $$\begin{array}{c} \frac{\left(TP+TN\right)}{\left(TP+TN+FP+FN\right)}\text{,} \end{array}$$

where TP represents the number of cases that are correctly classified as a nodule and TN represents the total number of cases that are originally not nodules but can be classified as a nodule. Negative classification cases which are also correct, FP represents the number of cases that are correctly classified as non-nodules. FN represents the number of cases that are originally nodules but can be classified as non-nodules.

The per-exam rates are also calculated for false positive and false negative; these measures are quite significant concerning performance measures in CAD evaluation because they depend equally on detection and classification.

The FP per exam rate is given by the following equation:

(7) $$\begin{array}{c} FE=\frac{FP}{n}\text{.} \end{array}$$

Here, *n* represents the number of exams used in tests. The FN per exam rate is given by the following equation:

(8) $$\begin{array}{c} FS=\frac{FN}{n}\text{.} \end{array}$$

### 3.11. Experimental Evaluation

20 CT scans have been collected from LIDC-IDRI which contains a total of 3592 slices. Each slice has a size of 512 × 512 pixels. There are in total of 738 nodules out of which 554 are non-nodules and 184 are nodules. The nodule size is in-between 3 mm to 30 mm. The pixel size is in-between 0.5 mm to 0.76 mm and the reconstruction interval ranges from 1 mm to 3 mm. We have distributed the dataset into training and testing datasets that have ranged from 20% training and 80% testing, 40% training, and 60% testing, 60% training, and 40% testing.

The article "An Efficient Model for Lungs Nodule Classification Using Supervised Learning Technique" was retracted in 2023. Reasons: signs of a paper mill; compromised peer review; unreliable results or conclusions.

### 3.12. Comparative Analysis

The comparison between the published CAD system and the proposed method is quite difficult because of the different datasets, nodule size, nodule type, and validation scheme. Here, the comparison between different CAD systems has been drawn based on two major factors these are dataset taken from LIDC and nodule size between 2 mm to 50 mm. The comparison has been presented in Table 3.

Comparisons in Table 3 demonstrate that the accuracy level of all techniques is below the proposed system except for the technique proposed by Ayyaz et al. [19], which is almost equal to the proposed technique; however, its false-positive rate is higher than the proposed technique. This shows that the proposed techniques outperformed the various existing techniques. In the proposed techniques, multiple thresholds were applied to remove non-nodule candidates which reduced the complexity of the system and also reduced the false positive rate.

## 4. Analysis and Discussion

Early and accurate detection of nodules helps to start the patient's treatment at an early stage and can reduce the mortality rate. About 80% of the patients who survive if malignancy is detected would be less than 20%. There are no chances of survival if the malignancy is detected at 75%. Lung malignancy detection is a complex process. During this study, it has been analyzed that several proposed techniques have the potential to perform well in the development of medical diagnostic tools. There were very few techniques that have high sensitivity with very few FPs per scan but normally increasing the sensitivity can cause a high rate of FPs. Table 3 demonstrates that the accuracy level of all techniques is below the proposed system except the technique proposed by Ayyaz et al. [19], which is almost equal to the proposed technique however its false-positive rate is higher than the proposed technique. This shows that the proposed techniques outperformed the various existing techniques. In this study, we have applied multiple thresholds so most of the non-nodules have been removed at earlier stages which can reduce system complexity as well as reduce FPs per scan. The overall system performance has been improved as shown in Table 3.

## 5. Conclusion

Most lung cancer cases are discovered at later stages, when it is more difficult to treat, which increases the mortality rate. Lung cancer screening at an early stage can greatly reduce mortality. Screening is a time-consuming process; therefore, CAD systems were created to aid radiologists in detecting lung nodules while minimizing diagnostic error and FPs rates. This study compared various supervised learning techniques for lung nodule identification and categorization. The taxonomy includes a full implementation of the most popular approaches as well as critical analysis. Based on prior methodologies, our proposed technique for detecting nodules and then classifying them using an SVM classifier has shown that the false positive rate (4 FPs/scan) is greatly reduced, with a sensitivity of 95%.

The article "An Efficient Model for Lungs Nodule Classification Using Supervised Learning Technique" was retracted in 2023. Reasons: signs of a paper mill; compromised peer review; unreliable results or conclusions.

## Figures and Tables

**Figure 1:** Proposed model.

**Figure 2:** (a) Original DICOM image. (b) Processed DICOM image.

**Figure 3:** (a) Lung volume after fixed thresholding. (b) Lung volume after applying morphological operation.

**Figure 4:** (a) Two big regions in lung volume. (b) After applying refinement and whole filling.

**Figure 5:** (a) Removing of critical section. (b) Intersection of segmented and original image.

**Figure 6:** (a) *B* & *W* to gray scale. (b) Refining of objects.

**Figure 7:** (a) Optimal thresholding byOstu method. (b) Rule-based pruning.

**Figure 8:** Steps from feature selection to classification.

**Table 1:** Pruning rules for nodule candidate detection.

Rule	Description
*R*1	Diameter < *T*_Min_*D*_
*R*2	Volume > *T*_Max_*V*_|elongation > *T*_*e*_|volume > *T*_Min_*V*_
*R*3	Diameter > *T*_Max_*D*_
*R*4	Circularity > *T*_*c*_ & area between *T*_Min_*A*_ & *T*_Max_*A*_

**Table 2:** Features for nodule detection.

Function index	Feature
2D geometric features	
*f*_1_	Area
*f*_2_	Diameter
*f*_3_	Perimeter
*f*_4_	Circularity
3D geometric feature	
*f*_5_	Volume
*f*_6_	Compactness
*f*_7_	Elongation
2D intensity-based statistical	
*f*_8_	Minimum
*f*_9_	Mean
*f*_10_	Variance
*f*_11_	Skewness
*f*_12_	Kurtosis
*f*_13_	Mean outside segment

**Table 3:** Performance comparison of CAD systems.

CAD system	Nodule size (mm)	Avg. FPs/scan	Sensitivity (%)
Murphy et al. [6]	<50	4.2	80.0
Wang et al. [9]	>10 and ≤20	1.19	69.3
Arnaud et al. [10]	3–30	4	90.1
Alex et al. [15]	2–10	1.17	90.6
Messay et al. [17]	3–30	3	82.66
Ayyaz et al. [19]	3–30	4.85	95.2
Proposed method	3–30	4	95

## Data Availability

The numeric data used to support the findings of this study are available from the corresponding author upon request.
